The article "Extra Dose of Vitamin C Based on a Daily Supplementation Shortens the Common Cold: A Meta-Analysis of 9 Randomized Controlled Trials" was retracted in 2023. Reasons: errors in the analysis; unreliable results or conclusions.

# Extra Dose of Vitamin C Based on a Daily Supplementation Shortens the Common Cold: A Meta-Analysis of 9 Randomized Controlled Trials

**DOI:** 10.1155/2018/1837634

**Published:** 2018-07-05

**Authors:** Li Ran, Wenli Zhao, Jingxia Wang, Hongwu Wang, Ye Zhao, Yiider Tseng, Huaien Bu

**Affiliations:** ^1^Graduate School, Tianjin University of Traditional Chinese Medicine, Tianjin 300193, China; ^2^Department of Neurology, Nankai Hospital, Tianjin Academy of Integrative Medicine, Tianjin 300100, China; ^3^Department of Research and Development, Hangzhou DeBuYou Health Technology Co. Ltd., Hangzhou, Zhejiang 310018, China; ^4^College of Traditional Chinese Medicine, Tianjin University of Traditional Chinese Medicine, Tianjin 300193, China; ^5^Department of Chemical Engineering, University of Florida, Gainesville, Florida 32611, USA

## Abstract

**Aim:**

To investigate whether vitamin C is effective in the treatment of the common cold.

**Method:**

After systematically searching the National Library of Medicine (PubMed), Cochrane Library, Elsevier, China National Knowledge Infrastructure (CNKI), VIP databases, and WANFANG databases, 9 randomized placebo-controlled trials were included in our meta-analysis in RevMan 5.3 software, all of which were in English.

**Results:**

In the evaluation of vitamin C, administration of extra therapeutic doses at the onset of cold despite routine supplementation was found to help reduce its duration (mean difference (MD) = -0.56, 95% confidence interval (CI) [-1.03, -0.10], and P = 0.02), shorten the time of confinement indoors (MD = -0.41, 95% CI [-0.62, -0.19], and P = 0.0002), and relieve the symptoms associated with it, including chest pain (MD = -0.40, 95% CI [-0.77, -0.03], and P = 0.03), fever (MD = -0.45, 95% CI [-0.78, -0.11], and P = 0.009), and chills (MD = -0.36, 95% CI [-0.65, -0.07], and P = 0.01).

**Conclusions:**

Extra doses of vitamin C could benefit some patients who contract the common cold despite taking daily vitamin C supplements.

## 1. Introduction

 The common cold, known simply as a cold, is defined as an upper respiratory tract infection (URTI) caused by various viruses, characterized by symptoms like coughing or sneezing, sore throat, stuffy or runny nose, headache, fever, muscle aches or aching limbs, and so on [1, 2]. However, because of similar symptoms, there is no way of distinguishing among the different types of common cold, other URTIs, and influenza in most cases.

With regard to virology and pathophysiology, URTIs are a group of diseases in the broad sense, including common cold, viral pharyngitis, laryngitis, herpangina, pharyngoconjunctival fever, and bacterial pharyngotonsillitis, rather than a single diagnosable disease [3]. About 70–80% of URTIs are caused by viruses, like rhinovirus, coronavirus, adenovirus, influenza and parainfluenza virus, respiratory syncytial virus, influenza A virus, and Coxsackie virus, and the other 20–30% are caused by bacteria [2, 4, 5]. Influenza is caused by the influenza virus, three subtypes of which affect humans (influenza viruses A, B, and C [6]); 30–80% of the cases of common cold have been attributed to over 200 strains of rhinoviruses [7, 8]. Influenza is highly contagious, with serious systemic symptoms and mild respiratory symptoms; its peak prevalence is in winter and spring; there are also global outbreaks and epidemics periodically [9–12].

The article "Extra Dose of Vitamin C Based on a Daily Supplementation Shortens the Common Cold: A Meta-Analysis of 9 Randomized Controlled Trials" was retracted in 2023. Reasons: errors in the analysis; unreliable results or conclusions.

As a frequently occurring acute upper respiratory tract disease, the common cold is self-limiting and generally lasts for 7–10 days or no more than 3 weeks [4]. The onset of the common cold is more acute, usually with nasal catarrh in the early stage. The common cold occurs in patients with low immunity, and the onset is seen year-round but more often in autumn, winter, and spring. The reason for the seasonality has not been conclusively determined. Further, people under great psychological stress [14] or undergoing intense training have a higher tendency to develop common colds [15, 16]. There are some reports stating that adults contract approximately 2 to 5 infections per year [17]; meanwhile, children develop common colds 6–10 times annually (up to 12 times among school children) [18]. The common cold does little harm on its own; however, it can be a serious complication when other diseases like pneumonia or meningitis develop comorbidly [19]. Despite rapid developments in science and medical technology, the common cold continues to pose a heavy burden worldwide, whether on human health or on economic losses. Fendrick AM et al. [20] reported that the economic burden attributed to the common cold in the US alone is US $40 billion annually (95% confidence interval (CI), $31.2–$48.0 billion). According to the data of the World Health Organization (WHO) from 2013, in America, the common cold accounted for 75–100 million physician visits per year at a conservative cost of US $7.7 billion per year, of which US $2.9 billion were for over-the-counter drugs and US $400 million were for prescription medicines. Additionally, an estimated 22 to 189 million school days were missed because of common colds, leading to 126 million missed workdays to look after children at home [21].

Because no effective therapies exist, treatment for the common cold is based on the relief of symptoms, including cough, sneezing, headache, fever, sore throat, and nasal congestion [21]. Current conventional symptomatic therapies are as follows: nasal decongestants; antihistamines (common cold may lead to a transient bronchial hypersensitivity; thus antihistamines are used); cough suppressants; nonsteroidal antipyretic analgesics, like aspirin; and expectorants. Additionally, identified in the early 1900s, in the search for the etiology of scurvy [22], vitamin C has been widely utilized in the prevention and treatment of the common cold or URTIs, with conflicting results with respect to its prophylactic effect. Some evidence has indicated that vitamin C could decrease the incidence of common cold and the duration of symptoms if taken regularly. Pitt et al. [23] found a reduction in the incidence of the common cold or associated morbidity among US Marines who were restricted to 2 g/day of vitamin C. In Constantini's study [24], vitamin C halved the duration of URTI episodes in male swimmers. More than 1 g/day of vitamin C shortened the duration of colds in adults by 8% and in children by 18% [25–28].

The article "Extra Dose of Vitamin C Based on a Daily Supplementation Shortens the Common Cold: A Meta-Analysis of 9 Randomized Controlled Trials" was retracted in 2023. Reasons: errors in the analysis; unreliable results or conclusions.

Inspired by the above-mentioned data, we conducted this meta-analysis to show whether vitamin C could be used for relieving symptoms, shortening the duration, or reducing the incidence of the common cold.

## 2. Methods

### 2.1. Search Strategy

The National Library of Medicine (PubMed), Cochrane Library, Elsevier, China National Knowledge Infrastructure (CNKI), VIP databases, and WANFANG databases were searched from their earliest records through March 2018 using the following key words: common cold, URTI [upper respiratory tract infection], vitamin C, and ascorbic acid. All the records were selected and screened by two independent reviewers, and a third reviewer was consulted when there was any disagreement. The review was conducted according to the guidelines for Preferred Reporting Items for Systematic Reviews and Meta-Analyses (PRISMA) [13].

### 2.2. Inclusive Criteria

#### 2.2.1. Study Type

We included randomized controlled trials (RCTs) related to the common cold using vitamin C as the therapeutic technique. Studies enrolled were reported in English or Chinese.

#### 2.2.2. Study Subject

Study subjects were those who were definitively diagnosed with the common cold based on laboratory examination, clinical signs, or reported symptoms. There was no limitation in age, sex, or occupation.

#### 2.2.3. Intervention

The intervention in the control group was a placebo, whereas the treatment group received vitamin C, which was added as a regular supplement or administered as needed when cold symptoms developed.

#### 2.2.4. Outcome

*(1) Efficacy Criteria. *The efficacy criteria were mean duration of the common cold (day); duration of main symptoms like nasal congestion or runny nose, sore throat, fever, aching in limbs and muscles, chest pain, chills, and mental depression (day); and socioeconomic impact (the days confined indoors).

*(2) Adverse Events. *If there were any abnormal signs and symptoms during treatment, adverse events would be discussed.

The article "Extra Dose of Vitamin C Based on a Daily Supplementation Shortens the Common Cold: A Meta-Analysis of 9 Randomized Controlled Trials" was retracted in 2023. Reasons: errors in the analysis; unreliable results or conclusions.

### 2.3. Exclusion Criteria

The exclusion criteria were duplicate articles; noninterventional studies, such as case-control study, cohort study, cross-sectional study, case reports and experiences, theory research, and reviews; nonclinical trials, such as animal testing; articles that assessed the use of vitamin C in the prevention of the common cold; and those in which vitamin C was used in the treatment group, with no placebo in the control group.

### 2.4. Quality Assessment

The quality of all trials was evaluated independently by two researchers, using the Cochrane collaboration's tool for bias risk assessment. The following items were assessed: random sequence generation, allocation concealment mechanism, blinding of participants and personnel, blinding of outcome assessment, incomplete outcome data, selective reporting, and other biases. The outcomes were evaluated as high risk, unclear, and low risk. Unclear was assigned if we could not find any descriptions of the item, low risk was assigned if the information was sufficient, and high risk was assigned if the information was inadequate.

### 2.5. Statistical Analysis

#### 2.5.1. Data Extraction and Synthesis

Pertinent dichotomous or continuous data were extracted and entered in the Review Manager 5.3 software for analysis. The risk ratio (RR) was used for dichotomous data, whereas the mean difference (MD) and standard deviations (SDs) were applied for continuous variables; for both, the corresponding 95% CI and forest plots were used. SD values were used when the data were in the same unit; and conversion should be made when different units were encountered in our meta-analysis.

#### 2.5.2. Data Conversion

Some trials provided the mean duration or severity of the common cold but not the SD. Under those circumstances, SD values were estimated when there was only sample size, median, range, or 95% CIs [38–40]. We calculated the SD value when the studies provided the standard error (SE) and mean values. Descriptive methods are used if the data are insufficient. Details are as follows:

① SDs were calculated if data on sample size and SE were available:
  (1) $$\begin{array}{c} SD=SE\times \sqrt{n} \end{array}$$
② Estimates of SD were calculated if sample size, mean, and 95% CI were available:
“a” is the upper confidence limit, and “b” is the lower confidence limit, so
  (2) $$\begin{array}{c} SD=\frac{a-mean}{1.96}\sqrt{n} \end{array}$$
or
  (3) $$\begin{array}{c} SD=\frac{mean-b}{1.96}\sqrt{n} \end{array}$$

The article "Extra Dose of Vitamin C Based on a Daily Supplementation Shortens the Common Cold: A Meta-Analysis of 9 Randomized Controlled Trials" was retracted in 2023. Reasons: errors in the analysis; unreliable results or conclusions.

#### 2.5.3. Assessment of Heterogeneity

Heterogeneity was detected by the Chi-squared test and* I*^2^ (inconsistency) statistics, with* P* < 0.10 or* I*^2^ > 50% indicating significant heterogeneity. As for our meta-analysis, when* P* ⩽ 0.05 or* I*^2^ > 50%, the random-effects model (DerSimonian-Laird method) was used, and the comparison was made between high-quality studies and the whole [41]; otherwise, the fixed-effects model was preferred.

## 3. Results

### 3.1. Study Selection

We identified 546 trials, and there were 423 records left after removing duplicates. Of those, 313 were in English, and the remaining 110 were in Chinese. We excluded 351 unqualified trials on the basis of titles and abstracts, and then 31 trials were excluded because of inappropriate contrast, while 32 were excluded for the assessment of prophylactic effect or other reasons. Finally, 9 articles [29–37] fulfilled our eligibility criteria after manual search and a review of full manuscripts. The study selection procedure is outlined in Figure 1.

### 3.2. Study Characteristics

A total of 9 trials [29–37] were included; they were randomized and controlled and included placebos. The 9 studies were from 1950 to 2001; 2 [30, 31] estimated the effect of vitamin C with supplementation at therapeutic doses, 4 [32–34, 37] estimated the therapeutic effect of vitamin C supplementation only at onset of the common cold, and the remaining 3 [29, 35, 36] assessed both. The principal characteristics have been summarized in Table 1.

### 3.3. Quality of the Included Studies

Table 2 reflected the quality of included studies with the risk of bias based on the Cochrane Handbook. All the studies were 100% completed and had no bias in selective reporting, but there was not any description to ensure whether other bias existed. Five studies [29–32, 36] mentioned random sequence, and 6 [29–34] mentioned allocation concealment. Except two articles [35, 37], the remaining 7 had low risk in blinding of outcome assessment and of participants and personnel. The study conducted by Lewib et al. [35] also had a low risk in blinding of participants and personnel.

### 3.4. Meta-Analysis of Outcome Criteria

#### 3.4.1. Mean Duration

The mean duration of the common cold was described in 9 trials, 2 of which were excluded in our meta-analysis, for the missing of SD or SE values [36, 37]. Displayed in Figure 2, there existed heterogeneity (Cochrane Q test = 31.78, df = 13, P = 0.003, and* I*^2^ = 59%), when the whole 7 trials were involved for analysis. Our meta-analysis was conducted on the random-effects model, with the result that vitamin C numerically shortened the duration of the common cold, but with no statistical significance (MD = -0.18, 95% CI [-0.67, 0.31], and P = 0.47). The results were different in the subgroup analysis; there was no significant effect (MD = 0.10, 95% CI [-0.64, 0.84], and P = 0.80) of vitamin C for treating the common cold if the patient was taking only therapeutic doses at the onset of illness. On the contrary, therapeutic doses of vitamin C at the onset of illness with regular supplementation shortened the common cold by about half a day (MD = -0.56, 95% CI [-1.03, -0.10], and P = 0.02).

The article "Extra Dose of Vitamin C Based on a Daily Supplementation Shortens the Common Cold: A Meta-Analysis of 9 Randomized Controlled Trials" was retracted in 2023. Reasons: errors in the analysis; unreliable results or conclusions.

There were 3 trials with relatively low quality [33–35]. With exclusion of the low-quality trials mentioned above, heterogeneity in total decreased (Cochrane Q test = 14.33, df = 8, P = 0.07, and* I*^2^ = 44%), whereas the result in total indicated an insignificant shortening of mean duration as before (MD = -0.07, 95% CI [-0.58, 0.43], and P = 0.78).

#### 3.4.2. Duration of the Main Symptoms

As shown in Figures 3–9, the main symptoms of common cold included nasal congestion or runny nose, sore throat, fever, aching limbs and muscles, chest pain, chills, and mental depression.

*(1) Nasal Congestion or Runny Nose. *With analysis on a fixed-effects model, the outcomes indicated that the vitamin C group had a better performance than did the placebo group as a whole, with no significance (MD = -0.02, 95% CI [-0.48, 0.43], and P = 0.92) and mild heterogeneity (Cochrane Q test = 9.04, df = 5, P = 0.11, and* I*^2^ = 45%). It seemed that the span of nasal congestion or runny nose was numerically decreased but not statistically significant (MD = -0.17, 95% CI [-0.78, 0.44], and P = 0.58), as the therapeutic doses of vitamin C after regular supplementation were given in the treatment group (Figure 3).

There was insignificant statistical difference (MD = -0.17, 95% CI [-0.78, 0.44], and P = 0.58) (Figure 3).

*(2) Sore Throat. *By conducting on a fixed-effects model, the days of sore throat pain in vitamin C group (regular supplemental plus therapeutic doses and therapeutic doses) were numerically fewer than those of placebo group but not statistically (MD = -0.26, 95% CI [-0.69, 0.16], P = 0.22) with no heterogeneity (Cochrane Q test = 2.42, df = 3, P = 0.49, and* I*^2^ = 0%) (Figure 4).

*(3) Fever. *According to the outcomes in Figure 5, the therapeutic doses after supplementation were significantly better at reducing fever by about half a day (MD = -0.45, 95% CI [-0.78, -0.11], and P = 0.009), showing no heterogeneity (Cochrane Q test = 0.01, df = 1, P = 0.90, and* I*^2^ = 0%).

*(4) Aching Limbs and Muscles. *As demonstrated in Figure 6, no matter the combination of supplemental and therapeutic doses of vitamin C (MD = -0.35, 95% CI [-0.70, 0.01], and P = 0.06) or therapeutic doses of vitamin C alone (MD = -0.02, 95% CI [-0.37, 0.33], and P = 0.92), there was no significant statistical difference from placebo group in aching limbs and muscles. There was no obvious heterogeneity (Cochrane Q test = 2.44, df = 3, P = 0.49, and* I*^2^ = 0%).

*(5) Chest Pain. *The symptom of chest pain was reported by Anderson et al. in 1975. Conducted on a fixed-effects model, the combination of supplemental and therapeutic doses of vitamin C significantly yielded a higher efficacy in relieving chest pain (MD = -0.40, 95% CI [-0.77, -0.03], and P = 0.03) with no heterogeneity (Cochrane Q test = 0.40, df = 1, P = 0.53, and* I*^2^ = 0%) (Figure 7).

*(6) Chills. *Because there was no heterogeneity (Cochrane Q test = 0.20, df = 1, P = 0.66, and* I*^2^ = 0%), the analysis was conducted on a fixed-effects model and proved that the combination of supplemental and therapeutic doses of vitamin C worked better at relieving chills by about 8 hours and a half (MD = -0.36, 95% CI [-0.65, -0.07], and P = 0.01) (Figure 8).

*(7) Mental Depression. *As is illustrated in Figure 9, supplemental and therapeutic doses of vitamin C could numerically reduce mental depression, but with no statistical significance (MD = -0.13, 95% CI [-0.49, 0.23], and P = 0.49) and heterogeneity (Cochrane Q test = 0.29, df = 1, P = 0.59, and* I*^2^ = 0%).

The article "Extra Dose of Vitamin C Based on a Daily Supplementation Shortens the Common Cold: A Meta-Analysis of 9 Randomized Controlled Trials" was retracted in 2023. Reasons: errors in the analysis; unreliable results or conclusions.

#### 3.4.3. Socioeconomic Impact: Being Confined Indoors

Because of mild heterogeneity (Cochrane Q test = 8.77, df = 5, P = 0.12, and* I*^2^ = 43%), the meta-analysis was conducted on a fixed-effects model. Some evidence revealed that vitamin C contributed to reducing about 6.5 hours of confinement indoors as compared to the placebo group (MD = -0.27, 95% CI [-0.46, -0.08], and P = 0.004). Particularly, therapeutic doses administered after daily supplements could reduce about 10 hours (MD = -0.41, 95% CI [-0.62, -0.19], and P = 0.0002) (Figure 10).

#### 3.4.4. Funnel Plot

Based on the mean duration of the common cold, funnel plot was applied to evaluate the publication biases of all 9 studies. Summarized in Figure 11, the outcome suggests that there was publication bias.

## 4. Discussion

### 4.1. Efficacy Analysis

Vitamin C (ascorbic acid), an essential nutrient found in fresh fruits and vegetables, is the most effective water-soluble antioxidant in human plasma. In the review by Hemilä H et al. in 2013 [27], therapeutic doses of vitamin C (0.2g/day or more) could shorten the duration of the common cold, but with no significance. Comparing with that, we could not come to the same conclusion (MD = 0.10, 95% CI [-0.64, 0.84], and P = 0.80), due to a strong heterogeneity like the differences of sex and dosage. Studies, respectively, conducted by Elwood PC [33] and Tyrrell DA [34] indicated that mere therapeutic doses of vitamin C were effective in males rather than females. It shortened the main duration (MD = -1.73/MD = -1.10), reduced the nasal congestion or running nose (MD = -0.69), and relieved the limb and muscle pain (MD = -0.11) in men. Given the sex differences in the effectiveness of the therapeutic doses of vitamin C, it is crucial to involve more intervention studies and to perform analysis based on gender or even age and intervention dosage.

The article "Extra Dose of Vitamin C Based on a Daily Supplementation Shortens the Common Cold: A Meta-Analysis of 9 Randomized Controlled Trials" was retracted in 2023. Reasons: errors in the analysis; unreliable results or conclusions.

As demonstrated by our meta-analysis comparing vitamin C with placebo, the combination of supplemental and therapeutic doses of vitamin C works on the common cold, while there is no statistically significant difference between mere therapeutic doses of vitamin C and placebo. To be specific, administration of extra doses of vitamin C at the onset of a common cold could help reduce the duration by about half a day (MD = -0.56, 95% CI [-1.03, -0.10], and P = 0.02), shorten the time confined indoors by about 10 hours (MD = -0.41, 95% CI [-0.62, -0.19], and P = 0.0002), and relieve the symptoms of a common cold, including chest pain (MD = -0.40, 95% CI [-0.77, -0.03], and P = 0.03), fever (MD = -0.45, 95% CI [-0.78, -0.11], and P = 0.009), and chills (MD = -0.36, 95% CI [-0.65, -0.07], and P = 0.01). Because there was no statistical heterogeneity in improving symptoms noted among the comparisons (all *I*^2^'s = 0%), we can safely conclude that vitamin C is therapeutic to some degree.

The efficacy mentioned above could help patients in shortening bad experiences and being earlier engaged in work. On account of this therapeutic effect, we would like to recommend a small daily dose of vitamin C (no more than 1.0g/day) to boost immunity and a larger dose of vitamin C during the common cold (a large dose than before, usually 3.0 g/day to 4.0 g/day) to better recover health.

### 4.2. Mechanism Analysis

In the 1960s, the American Nobel Laureate Linus Pauling stated in his book* Vitamin C and the Common Cold* that vitamin C could prevent and be used to treat the common cold. Immediately, this view spread globally. This concept is disputable and controversial, and there is a lack of sufficient evidence to support the use of vitamin C in the prevention and treatment of the common cold in the general population [42, 43]. Despite this, vitamin C is still widely administered during the common colds, and some evidence showed that it may reduce the duration of illness [27, 44]. The Swiss scientist Wintergerst E.S. [45] insists that because of its immune-enhancing effects vitamin C makes the body more capable of fighting off the virus, lessening the duration of the symptoms of the common cold. Vitamin C is concentrated in leukocytes, and its concentration rapidly declines during infections and stress. Vitamin C supplementation improves the ability to resist infection by improving the activities of the immune system, such as antimicrobial and natural killer cell activities, lymphocyte proliferation, chemotaxis, and delayed-type hypersensitivity [45]. Vitamin C also contributes to hormone regulation, including activation of the sympathetic nervous system and secretion of epinephrine during abnormal stress [46]. Additionally, vitamin C works at maintaining the redox integrity of cells and thereby protects them against the reactive oxygen species generated during respiratory burst and the inflammatory response [45].

The article "Extra Dose of Vitamin C Based on a Daily Supplementation Shortens the Common Cold: A Meta-Analysis of 9 Randomized Controlled Trials" was retracted in 2023. Reasons: errors in the analysis; unreliable results or conclusions.

### 4.3. Limitations

Although this study showed that vitamin C is beneficial, there were a few limitations associated with it. First, in some cases the data has to be calculated and transformed rather than being available directly. In some cases, the data were not suitable for a meta-analysis but were more suitable for a descriptive analysis because the 9 trials comparing vitamin C with placebo were relatively early trials. As a result, we eliminated several trials from our meta-analysis, weakening the exactness and representativeness of our data. Second, we were unable to recommend how many doses of vitamin C should be administered regularly and at the onset of a cold because there were no appropriate data (an obvious heterogeneity of the dosage before illness) to explore the dose-response relationship. Therapeutic RCTs must be conducted according to stricter, more precise guidelines to gain more knowledge on this subject. Finally, language limited our study and publication bias might result in inappropriate outcomes.

## 5. Conclusion

The combination of supplemental and therapeutic doses of vitamin C is capable of relieving chest pain, fever, and chills, as well as shortening the time of confinement indoors and mean duration.

## Figures and Tables

**Figure 1:** Study selection procedure. From [13].** For more information, visit www.prisma-statement.org.**

**Figure 2:** Forest plot of the meta-analysis of mean duration.

**Figure 3:** Forest plot of the meta-analysis of nasal congestion or runny nose.

**Figure 4:** Forest plot of the meta-analysis of sore throat.

**Figure 5:** Forest plot of the meta-analysis of fever.

**Figure 6:** Forest plot of the meta-analysis of aching limbs and muscles.

The article "Extra Dose of Vitamin C Based on a Daily Supplementation Shortens the Common Cold: A Meta-Analysis of 9 Randomized Controlled Trials" was retracted in 2023. Reasons: errors in the analysis; unreliable results or conclusions.

**Figure 7:** Forest plot of the meta-analysis of chest pain.

**Figure 8:** Forest plot of the meta-analysis of chills.

**Figure 9:** Forest plot of the meta-analysis of mental depression.

**Figure 10:** Forest plot of the meta-analysis of indoor confinement.

**Figure 11:** Funnel plot of publication bias in the comparison of vitamin C versus placebo.

**Table 1:** Characteristics of included studies in the comparison of vitamin C versus placebo.

**Author**	**Participants**		**Patients**		**Episodes of illness**		**Formulation**	**Dosing schedule**	**Outcome**
	**VC**	**P**	**VC**	**P**	**VC**	**P**			
**Anderson [29] 1974**	275	293	209	218	417	430	tablet	4g on the first day of illness	episodes of illness, duration, confined to house, off work
	305		231		483			8g on the first day of illness	
	277	285	212	233	436	437	tablet	1 g/d vitamin C and 4 g/d at onset of illness on the 1st day only	

**Anderson [30] 1972**	407	411	302	335	561	609	tablet	regular dose of 1g each day and increase to 4g each day for the first three days of any illness	episodes of illness, duration, confined to house

**Anderson [31] 1975**	150	146	Not reported	Not reported	Not reported	Not reported	tablet	500mg each week, 1500mg on the 1st day and 1000mg daily on days 2 through 5 during an illness	episodes of illness, duration, confined to house, off work, symptoms present
	152				Not reported		capsule		

**Audera [32] 2001**	47	42	47	42	Not reported	Not reported	tablet	1g/d at onset of illness for 3 days	duration, symptoms present
	50		50		Not reported		tablet	3g/d at onset of illness for 3 days	

**Elwood [33] 1977**	1082		32	33	Not reported	Not reported	tablet	3 tablets (3g) per day at onset of illness until the 10 tablets had been taken	duration
			39	25	Not reported	Not reported	tablet		

**Tyrrell [34] 1977**	724	777	225	257	*⩾*274	*⩾*329	tablet	4g/d for 2.5 days at onset of illness	duration, off work, symptoms present, in bed

**Lewis [35] 1975**	43	46	Not reported	Not reported	56	65	capsule	3g/d at onset of illness	episodes of illness, duration, side effect
	57		Not reported		76		capsule	regular dose of 3g each day and increase to 6g each day at onset of illness	

**Karlowski [36] 1975**	Not reported	Not reported	43	46	56	65	capsule	3g/d at onset of illness for 5 days	episodes of illness, duration, symptoms present
	Not reported		57		76		capsule	regular dose of 3g each day and increase to 6g each day at onset of illness	

**Cowan [37] 1950**	77	76	77	76	213	207	tablet	0.67 g of vitamin C every 4 hours at onset of illness, with a maximum of 10 doses	duration, severity

**Table 2:** Cochrane collaboration's tool for assessing risk of bias in the comparison of vitamin C versus placebo.

**Studies**	**Random sequence generation**	**Allocation concealment**	**Blinding of participants and personnel**	**Blinding of outcome assessment**	**Incomplete outcome data**	**Selective reporting**	**Other bias**
**Anderson [30] 1972**	low risk	low risk	low risk	low risk	low risk	low risk	unclear
**Anderson [31] 1975**	low risk	low risk	low risk	low risk	low risk	low risk	unclear
**Audera [32] 2001**	low risk	low risk	low risk	low risk	low risk	low risk	unclear
**Elwood [33] 1977**	unclear	low risk	low risk	low risk	low risk	low risk	unclear
**Tyrrell [34] 1977**	unclear	low risk	low risk	low risk	low risk	low risk	unclear
**Lewib [35] 1975**	unclear	unclear	low risk	unclear	low risk	low risk	unclear
**Karlowski [36] 1975**	low risk	unclear	low risk	low risk	low risk	low risk	unclear
**Cowan [37] 1950**	unclear	unclear	unclear	unclear	low risk	low risk	unclear

The article "Extra Dose of Vitamin C Based on a Daily Supplementation Shortens the Common Cold: A Meta-Analysis of 9 Randomized Controlled Trials" was retracted in 2023. Reasons: errors in the analysis; unreliable results or conclusions.

## Data Availability

All data are contained within the paper.

## Abbreviations

WHO: World Health Organization
PubMed: National Library of Medicine
CNKI: China National Knowledge Infrastructure
URTI: Upper respiratory tract infection
AURTI: Acute upper respiratory tract infection
PRISMA: Preferred Reporting Items for Systematic Reviews and Meta-Analyses
RCTs: Randomized controlled trials
SD: Standard deviations
RR: Risk ratio
CI: Confidence intervals
SMD: Standardized mean difference
SE: Standard error
MD: Mean difference.

## Supplementary Materials

Supplementary Materials PRISMA Checklist. PRISMA is an evidence-based minimum set of items for reporting in systematic reviews and meta-analyses. It focuses on the reporting of reviews evaluating randomized trials but can also be used as a basis for reporting systematic reviews of other types of research and particular evaluations of interventions.
